# Evaluation of the Antidiarrheal and Antioxidant Effects of Some Chewing Sticks Commonly Used for Oral Hygiene in Ghana

**DOI:** 10.1155/2021/7270250

**Published:** 2021-10-05

**Authors:** Edward Ken Essuman, Adjoa Agyemang Boakye, Clement Okraku Tettey, Gaston Hunkpe, Nii Korley Kortei, Henrietta Kwansa-Bentum, Sayanika Davi Waikhom, Enoch Aninagyei

**Affiliations:** ^1^Department of Nutrition and Dietetics, University of Health and Allied Sciences, Ho, Ghana; ^2^Department of Biomedical Sciences, University of Health and Allied Sciences, Ho, Ghana

## Abstract

Microbial etiology of diarrhea is a significant cause of death, especially in children in developing countries. The presence of microbes that are resistant to current treatment options for diarrhea suggests the need to find newer antimicrobial agents for treatment. Therefore, this study focused on investigating the antimicrobial effect of some Ghanaian chewing sticks commonly used for oral hygiene, *Azadirachta indica*, *Garcinia afzelii,* and *Garcinia kola*, against selected diarrhea-causing organisms. From the stem and bark of each plant, 70% methanolic extract was experimented on *Salmonella* and *Shigella* species, namely, *Shigella sonnei*, *Shigella flexeneri*, *Salmonella typhinirium enterica*, *Salmonella typhi* attenuated, and *Klebsiella oxytoca* for microbial susceptibility using the agar well diffusion method. Additionally, the antioxidant profile of the methanolic extracts were investigated using 2,2-diphenyl-1-picrylhydrazyl (DPPH) radical, 2,2'-azino-bis (3-ethylbenzthiazoline-6-sulphonic) acid (ABTS) scavenging activities, and ferric-reducing antioxidant potential (FRAP) assays, while the total polyphenolic content was determined using the Folin–Ciocalteau reagent. *G. afzelii* and *A. indica* stem demonstrated the highest antimicrobial effect, inhibiting the growth of all test organisms. Additionally, the extracts demonstrated high antioxidant potential and were found to possess significant amounts of phenolic compounds. Therefore, methanolic extracts of *G. afzelii* and *A. indica* stem are promising candidates for the identification of safe novel compounds to mitigate diarrheal diseases.

## 1. Introduction

Diarrheal disease is a significant global health problem that occurs in approximately 1.7 billion children yearly and is responsible for the death of around 525,000 children annually. After malaria, diarrheal disease is the leading cause of malnutrition in children less than five years of age and the second leading cause of mortality globally [1].

Diarrhea refers to a condition in which an individual may pass three or more liquid or loose stools per day. It occurs due to imbalances in the mechanisms regulating the secretion and absorption of water and electrolyte in the gut leading to dehydration [2, 3]. These imbalances can be caused by microorganisms (bacteria and viruses), helminths, toxins, diet, and allergic reactions [4]. Diarrheal disease is a medical emergency; hence, oral rehydration therapy, reduction in gut motility using antispasmodic drugs, and the use of antisecretory agents and drugs that inhibit secretion of prostaglandins, as well as antibiotic therapy, have proven to be very useful clinical interventions [5]. Despite the usefulness of these interventions in most cases, these therapies are not without discomforting side effects such as dry mouth, headaches, nausea, constipation, and drowsiness, which limit their usage [6, 7]. Additionally, a high prevalence of resistant strains of diarrheal pathogens has been observed in many developing countries where there is little restriction on the use of antibiotics and where the incidence of diarrhea-associated death in childhood is high [8, 9]. Hence, there is a need for the identification of newer therapeutic agents with fewer side effects and increased potency.

In developing countries, there is an increased reliance on natural product remedies for the management of both infectious and noninfectious diseases [10, 11]. Natural products are also seeing increased patronage even in the developed world [12]. In many African settings, these natural products are used to treat several medical conditions in folk medicine. These natural products have to be the source for the production of many orthodox medicines that are currently in use [11]. In 2012, Newman and Cragg reported that about half of the approved drugs over three decades were either directly or indirectly derived from natural products [13], due mainly to the high levels of phenol, alkaloid, saponin, and flavonoid secondary metabolites in such natural products [14]. Thus, investigating the ability of isolates from plant-based products to act as treatment options for different disease conditions is an important starting point in the search for newer therapeutic interventions for diverse disease states.

In Ghana, some selected roots, stems, and twigs of numerous plants have been used as chewing sticks for oral hygiene since time immemorial. Recent research has shown that these chewing sticks possess antimicrobial activity against selected oral disease-causing microbes such as *S. mutans, S. aureus,* and *E. coli* (unpublished data). Based on these observations and those from previously published results from Nigeria and Tanzania that these chewing sticks showed inhibitory effects against both Gram-positive and -negative bacteria [15, 16], we investigated the ability of these chewing sticks to exert inhibitory effects against common diarrhea-causing microbes since childhood diarrhea is still an important public health problem in Ghana [17]. Additionally, in bacteria-associated diarrhea, the microbial signals released by the infected microbes led to a substantive production of reactive oxygen and/or nitrogen species by the host to exert bactericidal effects on the infecting microbes [18]. These free radicals exert oxidative stress on the hosts by the lipid peroxidation mechanism leading to molecular damage and consequently tissue and organ failure, hence suggesting that therapeutic interventions that limit the production of these reactive species may prevent tissue damage induced by these enteric microbial infections. Some plant-based products are an important source of antioxidant molecules that scavenge for free radicals. Furthermore, the antibiotic properties of plant products cannot be overemphasized [19], thus making them an important target for finding therapeutic interventions for diarrhea and other enteric infections. This study aimed to carry out a preliminary investigation to determine if extracts from three commonly used chewing sticks in Ghana possessed any antimicrobial effects against selected diarrhea-causing bacteria as well as investigate the antioxidant potential of these isolates.

## 2. Materials and Methods

### 2.1. Study Plants and Preexperimental Preparations

The plants used in this study were *Azadirachta indica*, *Garcinia afzelii,* and *Garcinia kola.* For each plant, the stem and bark were used. Prior to obtaining the extract, the plant specimens were washed thoroughly with sterile distilled water. The washed plant specimens were air-dried for at least a month. The dried specimens were macerated into coarse pieces.

### 2.2. 70% Methanolic Extraction of Crude Plant Products

In a sterile conical glass jar, 2 L of 70% methanol solution was added to 200 g of each macerated plant sample. The plants samples were soaked for 48 hours with intermittent shaking. The methanol solvent filtrate was evaporated at 45°C in preweighed glass bottles in an oven.

### 2.3. Determination of Antimicrobial Activity

The test isolates, *Shigella sonnei* (DSM 5570), *Shigella flexneri, Salmonella typhi enterica* sub sp. *enterica* (ATCC19585), *Salmonella typhinirium* attenuated, and *Klebsiella oxytoca* (ATCC 13182), were obtained from the microbiology unit of the Department of Biomedical Sciences, University of Health and Allied Sciences. The agar diffusion method as previously used [20] and modified [21] was used. The test organisms were subcultured on Mueller-Hinton agar at 37°C between 18 and 24 hours. An inoculum (500 *µ*L) was adjusted to 1.5 × 10^8^ CFU/mL using 0.5 McFarland standard. On each Mueller-Hinton agar plate, each test organism was evenly spread using a sterile microbiological loop. The plate was incubated at room temperature (approx. 25°C) for 10 minutes. Subsequently, seven wells (diameter: 8 mm) were aseptically created into the agar medium. Into each of the wells, 100 *µ*L (5 mg/mL) of stems and backs of *Azadirachta indica*, *Garcinia afzelii,* and *Garcinia kola* extracts were aseptically dispensed into six individual wells while 30 *µ*L of a reference drug (chloramphenicol (CPL; concentration–5 mg/mL)) was dispensed aseptically into the seventh well. The Mueller-Hinton agar plates were incubated aerobically between 18 and 24 hours. The zones of inhibitions of the plant extracts were measured and compared to those of the reference drug.

### 2.4. Profiling of the Antioxidant Scavenging Activity of the Plant Extracts

The antioxidant activity of the study plants was evaluated using previously published protocols [22]. The antioxidant properties of the plant extracts were determined using the 2,2-diphenyl-1-picrylhydrazyl (DPPH) radical scavenging activity, 2, 2'-azino-bis (3-ethylbenzthiazoline-6-sulphonic) acid (ABTS) scavenging activity, ferric-reducing antioxidant potential (FRAP), and determination of total phenolic content.

#### 2.4.1. Determining DPPH Radical Scavenging Activity

The DPPH scavenging activity was determined by adding 200 *µ*L (mg/mL) of each plant extract to 800 *µ*L of 0.1 mmol/L of DPPH. The extract-DPPH mixture was incubated at room temperature for 30 minutes. Subsequently, the absorbance of the mixture was read spectrophotometrically at 517 nm using a VERSAmax microplate reader (Molecular Devices, San Jose, USA). Using the formula % scavenging [DPPH] = [(*A*_0_ − *A*_1_)/*A*_0_] x 100%, where *A*_0_ = the absorbance of the blank and *A*_1_ = the absorbance in the presence of the sample extract or standard (ascorbic acid), the % radical scavenging activity was calculated. Mean value from duplicate experiments was recorded. This protocol has been used in a recent study (Dravie et al., 2020).

#### 2.4.2. Determining ABTS Scavenging Activity

ABTS scavenging activity was determined by adding 200 *µ*L (mg/mL) of the plant extracts to 800 *µ*l of ABTS solution. The mixture was incubated at room temperature (25°C) for 10 minutes. Subsequently, the absorbance of the mixture was read spectrophotometrically at 734 nm using a VERSAmax microplate reader (Molecular Devices, San Jose, USA). The radical scavenging activity of the plant extracts was determined as recently published [22].

#### 2.4.3. The FRAP Assay

The FRAP assay was performed using the FRAP working reagent previously published [22]. In brief, 100 *μ*L (mg/mL) of the plant extracts was added to 3 mL of FRAP working reagent, incubated thermostatically for 30 minutes at 37°C. Using the VERSAmax microplate reader (Molecular Devices, San Jose, USA), the absorbance was measured at 593 nm. The absorbance of the plant extract corrected by the blank absorbance was proportional to the FRAP value. This protocol has been used in a recent study [22].

### 2.5. Estimation of Total Phenolic Content

The protocol for the determination of the phenolic content in the plant extracts has been published [22]. In brief, 0.5 g of the plant extract was dissolved in 5.0 mL methanol, followed by addition of 0.5 mL Folin–Ciocalteau reagent for 5 minutes. The mixture was incubated for 1 hour after adding 1 mL of 1 N sodium carbonate. The absorbance was read at 765 nm. Absorbance reading of each assay was converted to concentration using a calibration curve prepared using 100 *µ*g/mL, 200 *µ*g/mL, 400 *µ*g/mL, 600 *µ*g/mL, 800 *µ*g/mL, and 1000 *µ*g/mL solutions of gallic acid in methanol.

### 2.6. Data Analysis

Zones of inhibition of plant extracts were measured in millimeters and compared to those of the reference drug. Data were presented as mean ± SEM. Tabular and graphical presentation were used to present data.

## 3. Results

Analysis of zones of inhibition indicated that the microorganisms examined were susceptible to *G. afzelii* and *G. indica* stem, whereas none of the microorganisms examined except for *S. sonnei* was susceptible to *G. kola* stem. *G. kola* and *A. indica* barks displayed no antimicrobial activity against *S. typhimurium enterica.* Additionally, the *A. indica* stem did not inhibit the growth of *S. flexneri* (Table 1).

The extracts demonstrated significantly high DPPH radical scavenging activity (Figure 1). Both *A. indica* stem and *G. kola* bark exhibited the highest DPPH radical scavenging effect, which was as high as 89.58%. This was followed by *G. afzelii* stem (87.08%), *A. indica* bark (86.25%), *G. kola* stem (85.00%), and *G. afzelii* bark (81.25%). The ascorbic acid standard recorded 94.17% inhibition (Figure 1).

The extracts used in this study were found to quench ABTS free radicals significantly in a manner comparable to the ascorbic acid standard (98.83%) (Figure 2). *G. kola* stem demonstrated the highest activity by scavenging about 99.53% ABTS radicals. This was followed by *G. afzelii* stem and *G. kola* bark (99.30%), *A. indica* bark (99.06%), *G. afzelii* bark (98.12%), *A. indica* stem (96.01%).

Furthermore, extracts from the chewing sticks examined in this study demonstrated exceedingly high FRAP values (Table 2). The highest FRAP value was recorded for *A. indica* bark (2.29 ± 0.15). This was followed by *G. afzelii* bark (2.24 ± 0.05), *G. kola* bark (1.85 ± 0.15), *G. afzelii* stem (1.64 ± 0.18), *G. kola* stem (1.61 ± 0.01), and *A. indica* stem (1.26 ± 0.07).

Except for the *A. indica* stem, all extracts demonstrated appreciable total phenolic contents in gallic acid equivalence (GAE) (Figure 3). The highest phenolic content was observed in *G. afzelii* bark extract (75.38 µgGAE/g), followed by *G. kola* bark (71.93 µgGAE/g), *G. afzelii* stem (68.15 µgGAE/g), *A. indica* bark (67.28 µgGAE/g), *G. kola* stem (62.67 µgGAE/g), and *A. indica* stem (30.33 µgGAE/g).

## 4. Discussion

Due to the increasing prevalence of antibiotic resistance and the toxicity associated with synthetic drugs products, several studies have attempted to find plant products with antimicrobial properties due to their tolerability on the body. In this study, the antimicrobial effects of methanolic extract of three different plants, namely, *Azadirachta indica*, *Garcinia afzelii,* and *Garcinia kola*, commonly used as chewing sticks in Ghana for oral hygiene against some diarrhea-causing pathogens are evaluated. These organisms included two *Shigella* spp., *S. sonnei* and *S. flexneri*, which have been associated with shigellosis with symptoms of diarrhea, fever, vomiting, and stomach cramps. Worldwide prevalence of shigellosis is 164.7 million people annually, with greater than 95% of the cases occurring in developing countries [23]. Antimicrobial effects on other microorganisms such as *Salmonella typhi enterica, Salmonella typhinirium* attenuated*, L. innocua, and K. oxytoca* which have been associated with different forms of diarrheal diseases in the literature were also examined [24–26].

Our results showed that *G. afzelii* and *A. indica* stem inhibited the growth of the entire microorganism examined to varying degrees using the agar well diffusion assay. In a related study, a similar inhibitory effect of *G. afzelii* and *A. indica* stem against S. *aureus* and *E. coli* was observed (*unpublished data*). These two microbes have also been associated with diarrhea [27, 28]. *G. kola* stem showed the least antimicrobial activity inhibiting the growth of only one of the *Shigella* species.

Since all extracts demonstrated antibacterial effects to various extents, it can be concluded that each chewing stick sample may possess various inhibitors of bacteria, hence the observed biological activities. Previously, Ashie et al. [29] investigated the microbial pathogens associated with acute childhood diarrhea within a Ghanaian setting, and *Salmonella* spp. and *Shigella* spp. were found to be the most prevalent bacterial species associated with diarrhea. Our results showing an inhibitory effect of the chewing stick extracts on these two microbes as well as other diarrhea-causing microbes is, therefore, of important public health consequence since it may lead to the potential isolation of bioactive compounds that can be used in the treatment of diarrhea.

Antioxidants are molecules that scavenge free radicals and are important for maintaining good health. In response to an infected microbe, the body releases a host of reactive oxygen and nitrogen species to fight the infection; however, excessive production of these free radicals can result in tissue damage which leads to other complications [18]. Maintaining a good balance of oxidants and antioxidants is very essential for maintaining enteric health. The results of the present study reveal that the chewing stick extracts possess exceptionally high antioxidant effects in both the DPPH and the ABTS assays.

The 2,2-diphenyl-1-picrylhydrazyl (DPPH) is a known nitrogen-centred free radical. Therefore, any products with adequate antioxidant activity can scavenge for a significant amount of this radical and, hence, may be useful to reduce oxidative stress in organisms. We demonstrated that all the plant extracts were able to significantly reduce the initial amount of the DPPH free radical in the solution. One attribute of antioxidants is to scavenge for proton radical [30]. Therefore, continuing usage of these plants as chewing stick could reduce oxidative stress in humans. Additionally, these plants could provide useful compounds for formulation of antioxidants for human use. Furthermore, the initial level of 2, 2'-azino-bis (3-ethylbenzthiazoline-6-sulphonic) acid (ABTS) scavenging activity was reduced by the plant extracts. This cationic radical is able to react with most antioxidants to reduce their bioavailability *in vivo* [31].

In this experimental study, we investigated the transformation of ferric (Fe^3+^) to ferrous (Fe^2+^) iron as a measure of the reductive potential of the various extracts. Again, all extracts used in this study demonstrated significant ferric iron-reducing antioxidant potential. This potential makes the strong antioxidants [32]. Reducing properties have been linked to the presence of reductone, which demonstrates antioxidant properties by breaking chain reactions and are also potent inhibitors of peroxide formation. Some peroxides such as H_2_O_2_ have been linked to tissue injury and cell toxicity, and hence, there is a need to adequately control their levels by reduction. From our results, the exceptionally high antioxidant effects demonstrated by the various chewing sticks present them as candidates for the extraction of novel antioxidant compounds.

We also found out that the plant extracts contain high levels of phenolic compounds. Meanwhile, most of the antimicrobial properties of plants are attributed to phenol and flavonoid secondary metabolites. Also, phenols have been shown to exhibit strong antioxidant activity [33]. Taken together, *G. afzelii* and *A. indica* have been found to inhibit the growth of *S. sonnei*, *S. flexeneri*, S*. typhinirium enterica*, *S. typhi* attenuated, and *K. oxytoca* and, hence, may reduce incidences of diarrhea when chewed continually. Additionally, these plants were found to possess high antioxidant activity. Therefore, even though these plants are chewed for the purses of oral hygiene, users may unknowingly be protecting themselves from diarrhea-causing pathogens and, at the same time, neutralizing free radicals in the body. These properties of the plants are important for maintaining better human health and preventing diseases.

## 5. Conclusions

Our results show that *A. indica* and *G. afzelii* stem, which are commonly used chewing sticks in Ghana, possess potent antimicrobial activity against common diarrhea-causing microorganisms. All extracts examined also contained significant antioxidant activity. The high phenolic content of the plants may be responsible for the high antioxidant and potent antimicrobial activities observed in the study. These chewing sticks, therefore, can be further studied in the future to elucidate the actual compound producing the observed biological activity. Finally, the continual use of these plants for oral hygiene must be encouraged.

## Figures and Tables

**Figure 1:** DPPH scavenging activity of chewing stick extracts and standard ascorbic acid.

**Figure 2:** ABTS radical scavenging activity of chewing stick extracts and standard ascorbic acid.

**Figure 3:** Total phenolic contents of chewing stick extracts.

**Table 1:** Antimicrobial activity of chewing stick extracts against selected microorganisms.

Organism	Zone of inhibition (mm)						
	*A. indica*		G. *afzelii*		*G. kola*		CPL
	Stem	Bark	Stem	Bark	Stem	Bark	
*S. sonnei* (DSM 5570)	13	4	10	12	3	9	24
*S. flexneri*	14	0	18	16	0	11	19
*S. typhi*	9	14	10	13	0	11	29
*S. typhimurium enterica* sub sp. (ATCC19585)	15	0	12	19	0	0	28
*K. oxytoca* (ATCC13182)	15	8	13	14	0	14	31

**Table 2:** Mean FRAP values of chewing stick extracts compared to standard ascorbic acid.

Samples	*A. indica* stem	*A. indica* bark	*G. afzelii* stem	*G. afzelii* bark	*G. kola* stem	*G. kola* bark	Ascorbic acid
Mean FRAP value	1.26 ± 0.07	2.29 ± 0.15	1.64 ± 0.18	2.24 ± 0.05	1.61 ± 0.01	1.85 ± 0.15	2.00 ± 0.00

## Data Availability

All data are in the manuscript.
